# Double-UV Photoionizaion Detector with Graphene Oxide-Coated Electrodes

**DOI:** 10.1155/2022/4330518

**Published:** 2022-07-19

**Authors:** Qi Zhou, Xu Zhang, Xu Ma, Sixiang Zhang

**Affiliations:** ^1^School of Electrical Engineering and automation, Tianjin University of Technology and Education, Tianjin 300222, China; ^2^Tianjin Key Laboratory of Information Sensing and Intelligent Control, Tianjin 300222, China; ^3^School of Mechanical Engineering, Tianjin University of Technology and Education, Tianjin 300130, China; ^4^School of Electrical and Electronic Engineering, Tianjin University of Technology, Tianjin 300130, China; ^5^School of Mechanical Engineering, Hebei University of Technology, Tianjin 300130, China

## Abstract

The structure of a photoionization detector was optioned and researched. In order to solve the problem of the photoionization detector' lamp surface residue interference, a new structure of the self-cleaning double-UV detector was adopted. At the same time, the air flow field of the detector was simulated by the finite element method. Through analyzing the results of the simulation experiment, further optimization of the gas channel for the microdetector was carried out, and the ionization chamber with axial flow structure was finally chosen. The new nanomaterial, graphene oxide was used to modify the surface of the collector plate of detector to improve the gas sensitivity and sensitivity of the photoionization detector. Through the experimental analysis, the performance indexes of detector were described in detail. The minimum detection limit of the detector is 2.5 × 10^−7^. The linearity response of the detector was analyzed, and the linear correlation coefficient reaches 0.993. The experimental results show that the double-UV detector can improve the overall gas sensing characteristics and provide an ideal detection unit for volatile organic compound (VOC) gas detection.

## 1. Introduction

Volatile organic compounds (VOCs) is an important part of air pollution and an important index of quantitative air pollution. The boiling point of VOCs gas is 50°C-260°C, and its saturated vapor pressure usually exceeds 133.32 Pa at room temperature. According to its chemical structure, VOCs gas can be roughly divided into alkanes, aromatics, esters, aldehydes, and so on [1, 2]. They exist widely in the atmosphere, water, and soil. On the one hand, they cause serious pollution to the environment [3]; on the other hand, they seriously endanger people's physical and mental health. Therefore, the detection of VOCs gas is particularly important in environmental protection. This paper mainly researches photoionization detector (PID) [4], which is the core component of VOCs gas detection, as the main object to carry out the theoretical and experimental research.

According to the requirements of VOC detection, a micro-PID was fabricated using MEMS technology. Different types of microchannel were designed. The effects of different physical and chemical parameters were experimentally investigated. The key parameters affecting the efficiency of microchannel such as carrier gas pressure [5], temperature, and flow rate, were experimentally investigated.

Graphene belongs to the category of two-dimensional materials, which has significant advantages in specific surface area and physical adsorption compared with activated carbon. In the laboratory, this material is generally obtained by chemical vapor deposition and other methods. Graphene oxide (GO) has a large specific surface area, but its structure is imperfect compared with intrinsic graphene, which is mainly reflected in unpaired electrons, so it is likely to combine with gas molecules [6]. Besides, there are many oxygen-containing functional groups in the microstructure of GO, which is the reason why it has a large specific surface area and strong adsorption capacity. Therefore, graphene has great room for development in the field of VOCs. It can greatly enhance the gas sensing properties of the plate surface by introducing graphene into the electrode of PID.

## 2. Materials and Methods

There is an ultraviolet light as the ionization source to ionize the gas molecules of the material in photo ionization detector. During the working process of PID, the inert gas in the UV lamp of PID is excited in the alternating high frequency electric field to form a plasma. Through releasing photons, the gas to be measured is ionized [7]. Therefore, the reaction in the ionization chamber has a great influence on the photocurrent produced by photoionization. Its ionization efficiency directly affects the determination of gas concentration by photoionization detector.

The traditional single-lamp PID detector is basically divided into one-dimensional structure and two-dimensional structure. Axial flow (Figure 1(a)) shows orthogonal relation between UV lamp path, gas path, and collecting plate, and the gas path diameter is determined to be 1.2 mm, and the electrode width is 1 mm [8, 9]. In order to improve ionization efficiency of photoionization detector for gas and to solve the problem of self-cleaning of the lamp surface, a new structure—dual-lamp PID detector—is presented. The comparison between the single-lamp and dual-lamp detector structures is shown in Figure 1.

The traditional PID sensor with single-lamp structure adopts three-dimensional orthogonal structure, and the gas is not in direct contact with the UV lamp, which improves the pollution of the lamp surface because of long-term use to a certain extent. However, when detecting sulfide and other easily adsorbable gases for a long time, the baseline will rise and the response will drop. When the ionization potential is close to the ionization energy of the UV lamp, the ionization efficiency decreases obviously. The dual-lamp structure adopts the structure of two UV lamps facing each other. On the one hand, the problem of cleaning the lamp surface can be improved. On the other hand, the luminous efficiency of the UV lamp can directly affect the performance of the sensor. But the effective spectral lines are few, therefore, the ionization efficiency can be increased when detecting gases with higher ionization potentials.

After determining the structure of the dual-lamp PID, the structure of the gas path in the ionization chamber is further optimized by simulation experiments [10]. The structure of the ionization chamber is shown in Figure 2(a)). Due to the larger volume of the rectangular ionization region of the sensor and the smaller size of the gas inlet, the convex structure will be formed when entering the ionization region. Therefore, the gas circuit structure has been improved. As shown in Figure 2(b)), the internal gas circuit structure of the sensor has been processed by the overimprovement of the cone to reduce the abrupt change in the cross-sectional area of the gas circuit structure inside the ionization chamber and ensure the interior of the ionization chamber, which ensures the internal volume of the ionization chamber and also ensures the performance of the sensor.

Through theoretical analysis and experiments, we know that when a rectangular plate is used to excite the UV lamp, the UV lamp emits a linear beam perpendicular to the two electrode plates. When a ring plate is used to excite the UV lamp, the lamp emits a cylindrical beam, and its diameter is approximately the same as the diameter of the lamp. The available area of the beam is large so that the gas to be measured in the chamber will be entirely exposed to ultraviolet light. Hence, a strong current signal is generated, the efficiency of the UV lamp is improved, and the difficulty of detecting the current signal is reduced. Therefore, gas circuit simulation results are used in the channel design, which is shown in Figure 3.

When the electrostatic field is an electric field, the calculation expression of the electric potential energy of neutral polarizable molecules is −*αE*(*r*)^2^/2 [11], where *α* represents the static molecular polarizability, *r* represents the position of the molecule, and *L* and *K* represent the radial and axial momentum between the molecule and the plate, respectively. From this, a dependency of the inverse square is determined. The effective electric potential energy obtained by its radial motion is [12]

(1) $$\begin{array}{c} U_{r}\left(r\right)=\frac{L}{2{mr}^{2}}-\frac{K^{2}}{2{mr}^{2}}. \end{array}$$

According to the above formula, two different ion motion models can be judged, which are closely related to the size of *L* and *K*. In the case of *L* > *K*, the molecule is finally captured by the graphene oxide layer because the polarization is greater than the radial potential energy. Otherwise, when *L* < *K*, the motion phenomenon of repulsive radial potential energy caused by the eccentric potential energy will occur, so we can draw a conclusion that whether molecules will be captured by the plates depends on the voltage between the plates, which indirectly determines the efficiency of plate ionization. Then, the probability formula of electron tunneling ionization in a strong field [13] is derived from the Ammosov-Delone-Krainov model, that is, the ionization efficiency formula of gas:

(2) $$\begin{array}{c} W_{a}\left(E\right)=\frac{4^{n}\xi_{1}}{n^{*}\Gamma \left(2n^{*}\right)}{\left(\frac{2\xi_{0}}{E}\right)}^{2n^{m}-1}\exp\left(-\frac{2\xi_{0}}{3E}\right), \end{array}$$

where *W*_*a*_ is the gas ionization efficiency, *E* is the electric field strength, and *ξ*_1_ is the ionization energy required for gas ionization. Because the ionization energy is determined by the type of gas, the gas ionization efficiency is only related to the intensity of the electric field. The higher the voltage, the higher the ionization efficiency. The response mechanism of PID based on graphene oxide as the collector to gas is to use the electric field formed by the position of the nanotip. This tip effect combines with electric field, which can enhance microcurrent response obviously under equal voltage condition, thus improving gas sensing properties. Therefore, this method is beneficial to gas detection [14, 15].

## 3. Results and Discussion

A mass flow controller (MFC) was used to adjust pump suction flow, and volume flow is set to 50 mL/min [16], when the system is stable and the background gas is relatively stable. Low-concentration injection (toluene with a volume fraction of 500 ppb for single-lamp sensor and dual-lamp sensor) was carried out, respectively [17]. After processing response through microcurrent amplifier and then collecting after I/V conversion, the specific results are shown in Figure 4.

Voltage response value of dual-lamp sensor is *V*_1_ = 0.73 V, and voltage response value of single-lamp sensor is *V*_2_ = 0.57 V. Response margin is Δ*V* = 0.16V. Through experiments, it was found that after low concentration gas detection, the baseline drift of a single-lamp sensor is significantly more serious than that of a dual-lamp sensor, and the required baseline stabilization time is longer than that of a dual-lamp sensor. After the baseline returns to zero and stabilizes, high-concentration injections (toluene with a volume fraction of 2 ppm) were performed for the single-lamp sensor and the dual-lamp sensor, respectively. Experimental results are shown in Figure 5.

The voltage response value of dual-lamp sensor is *V*_1_ = 2.41 V and that of single-lamp sensor is *V*_2_ = 2.09 V. The response difference is Δ*V* = 0.32V. It can be seen that the performance of dual-lamp sensor is better than that of single-lamp sensor in a wide range (volume fraction is 500 ppb-2 ppm). And it can obviously improve the interference caused by the lamp pollution of the sensor.

The principle of chemical oxidation is to treat (intercalate and oxidize) graphite with a strong oxidant to obtain graphite oxide. The microstructure of this product has functional groups with good hydrophilicity, so that effect of the layers inside the graphite is reduced. Therefore, the strong oxidant can destroy the van der Waals force between each layer of graphite and then make each layer independent. The single-layer graphite oxide obtained in the above process is placed in an ultrasonic environment, separated by an organic solvent, and finally reduced to a single layer. The layered graphene [18] is dissolved in the solution and diluted to a 1 mg/mL graphene oxide solution, which is convenient for subsequent operation and treatment. Then, the Cu electrode was soaked in PEG solution of 5 mmol/L for 12 hours [19] and dried and soaked in graphene oxide solution for 5 hours. The amino group in the PEG solution [20] was combined with the carboxyl group in graphene oxide solution to make graphene oxide adhere to the surface of the plate. According to the different soaking times, the graphene oxide electrodes [21, 22] soaked for 1 time, 2 times, and 3 times were detected, respectively, with 500 ppb isobutene gas. It is concluded that the graphene oxide-covered electrode can effectively improve the gas sensing properties of the sensor, and the graphene oxide on the surface of the plate will combine more fully with the increase of soaking times. The voltage response value is shown in Figure 6.

## 4. Conclusions

In this article, the influence of single-lamp and dual-lamp on the signal of PID based on the principle of photoionization was mainly discussed, and the sensor plate was optimized by new nanomaterials. According to the principle model of the sensor, a complete dual-light ionization sensor structure model was established. Through the analysis of the comparative experimental results of high and low concentration toluene, the performance improvement of the new PID was verified. The graphene oxide electrodes with different immersion times were tested with 500 ppb isobutene, and the electrode parameters and properties were determined, which provides a reliable data basis and experience for the follow-up work. It is inferred from the experiment that there is a good linear relationship between the voltage response and the concentration of PID for toluene in the measurement range of 0 ppm-8 ppm, and the lowest detection limit is 250 ppb. It is concluded from the experiment that the voltage response and concentration of toluene PID have a good linear relationship in the measurement range of 0 ppm-8 ppm, and the minimum detection limit is 250 ppb.

## Figures and Tables

**Figure 1:** The PID detector structure.

**Figure 2:** The whole gas path model.

**Figure 3:** Gas circuit simulation results.

**Figure 4:** Single lamp-double light sensor response for 500 ppb.

**Figure 5:** Single lamp-double light sensor response for 2 ppm.

**Figure 6:** Voltage response contrast of the graphene oxide-coated electrode sensor with different soaked times.

## Data Availability

No data were used to support this study.
